The article "Multidrug-Resistant Bacteria: Their Mechanism of Action and Prophylaxis" was published in 2022. Journal: Biomed Res Int.

# Multidrug-Resistant Bacteria: Their Mechanism of Action and Prophylaxis

**DOI:** 10.1155/2022/5419874

**Published:** 2022-09-05

**Authors:** Alok Bharadwaj, Amisha Rastogi, Swadha Pandey, Saurabh Gupta, Jagdip Singh Sohal

**Affiliations:** Department of Biotechnology, GLA University, Mathura (U.P.)-281 406, India

## Abstract

In the present scenario, resistance to antibiotics is one of the crucial issues related to public health. Earlier, such resistance to antibiotics was limited to nosocomial infections, but it has now become a common phenomenon. Several factors, like extensive development, overexploitation of antibiotics, excessive application of broad-spectrum drugs, and a shortage of target-oriented antimicrobial drugs, could be attributed to this condition. Nowadays, there is a rise in the occurrence of these drug-resistant pathogens due to the availability of a small number of effective antimicrobial agents. It has been estimated that if new novel drugs are not discovered or formulated, there would be no effective antibiotic available to treat these deadly resistant pathogens by 2050. For this reason, we have to look for the formulation of some new novel drugs or other options or substitutes to treat such multidrug-resistant microorganisms (MDR). The current review focuses on the evolution of the most common multidrug-resistant bacteria and discusses how these bacteria escape the effects of targeted antibiotics and become multidrug resistant. In addition, we also discuss some alternative mechanisms to prevent their infection as well.

## 1. Introduction

In the present situation, an increase in antibiotic-resistant microorganisms has become one of the most vital threats to the healthcare sector. Multidrug-resistant bacteria (MDR) that are deadly pathogenic are rising day by day and pose a very serious threat to human health. Earlier, these types of antibiotic-resistant bacterial strains were rare and limited to only nosocomial-acquired infections, but nowadays, they have become very common. This issue is more prevalent among both Gram-positive and Gram-negative bacterial species, which include *A. baumannii*, *E. coli*, *P. aeruginosa*, and *K. pneumonia* (Gram-negative), along with *S. aureus*, *S. pneumoniae*, *E. faecium*, and *E. faecalis* (Gram-positive). It has been found that this antibiotic resistance occurred among these bacterial species due to the attainment of plasmids through the transfer of resistance genes [1]. To escape from the harmful effects of antibiotics, certain bacterial species develop some special mechanisms like efflux pumps, less permeability of the LPS layer, secretion of degrading enzymes, and alteration of targets [2]. Certain factors that are responsible for increasing this antibiotic resistance may include widespread development, overexploitation of antibiotics, extreme use of broad-spectrum drugs, and scarcity of target-oriented antimicrobial drugs [3].

The article "Multidrug-Resistant Bacteria: Their Mechanism of Action and Prophylaxis" was published in 2022. Journal: Biomed Res Int.

## 2. Community, Nosocomial, and Healthcare-Associated Infections

Initially, MDR bacteria were associated with hospital-acquired infections. MDR bacteria have spread and are now the leading cause of community-acquired infections. The spread of multidrug-resistant (MDR) bacteria in society has resulted in an increase in morbidity, mortality, healthcare expenditure, and antibiotic use. According to the IDSA (the Infectious Diseases Society of America), resistance to antimicrobial compounds can be defined as “one of the greatest threats to human health worldwide” [4]. It has been observed that patients infected with MDR strains of bacteria have more severe consequences than patients infected with other vulnerable organisms [5, 6]. As a result, this increase in the spread of antibacterial resistance leads to posing a serious threat to society as well as to the medicines available and also causes a negative impact on cancer therapy, transplantation, and surgical events [7]. It has been assumed that the occurrence of particular MDR bacterial strains is strongly associated with the application of broad-spectrum antibiotics that consist of empiric along with definitive therapy [8]. Such overexploitation is responsible for the higher incidence of MDR and leads to the development of a vicious cycle.

Infection is an ill-state and could be classified into two types: society-associated and nosocomial. Differentiation among two types of infections is based on whether the beginning of illness was up to the first two days of hospitalization (community-associated) or afterwards (nosocomial type). As per the work initiated by Morin et al. and Friedman et al., community-associated infections can be further classified into healthcare-associated and community-acquired infections [9, 10]. If the patient was in a hospital under critical care for 48 hours or more; within 90 days of the infection; admitted to the hospital or persistent care for an extended period of time; received chemotherapy; intravenous antibiotic treatment; or wound care in the previous month of the existing illness [11], this is considered a healthcare-associated infection. On the other hand, community-acquired infections consist of those patients having a community-onset infection along with those who do not match the above criterion (healthcare-associated infection). Though such criteria are capable of solving and accessing the spread of MDR bacteria in society, they are not enough to explain the complete story. It has been observed that the patients get infected with the same organism with which they were colonized earlier. Henceforth, the moment of colonization is more significant in comparison to the moment of infection diagnosis as far as the origin of MDR bacteria is concerned.

The article "Multidrug-Resistant Bacteria: Their Mechanism of Action and Prophylaxis" was published in 2022. Journal: Biomed Res Int.

## 3. Transitioning from a Hospital-Acquired Pathogen to a Society-Associated Pathogen

It has been noticed in various studies that the frequent use of antibiotics always becomes a threat to mankind. The increase in antibacterial resistance patterns can vary according to the threat associated with the particular antibiotic class. Here, an attempt has been made to explain the link between the application of a particular antibacterial agent and the origin of resistance to a specific antibiotic. The application of tigecycline to individuals suffering from *Klebsiella pneumonia* containing carbapenem-resistant infection was observed to develop tigecycline resistance in the same bacterial strain, which was a very crucial example [12]. From this instance, it has become evident that we have to manage and control this antibacterial resistance in all aspects, i.e., at the level of nosocomial infections, societal level infections, and nonmedical antibiotics. Moreover, healthcare devices pose a supplementary risk factor for multidrug-resistant bacteria. Certain medical devices, like endotracheal tubes, urinary catheters, vascular lines, and feeding tubes, are also recognized as high-risk factors [13]. In addition to it, other risk factors responsible for the illness or establishment of multidrug-resistant bacteria may include immunocompromised conditions like transplantation of any organ or hematopoietic stem cell along with other factors like kidney failure [14]. Among the microorganisms, such resistance genes are found to be beneficial for the organism and have implausibly spread in society, except when the compensatory genetic material is collected or through the application of antibiotics, the expression of the resistance gene gets completely induced. One good example of such an event is erythromycin resistance methylase (erm) genes that act as inducible genes and are present in *S. aureus* and *Mycobacterim.* Such genes are expressed only when the bacteria are treated with the particular antibiotic that results in the development of antibiotic resistance among the bacteria.

Among the bacterial community, the development of biofilm is a unique characteristic of their life cycle. The formation of biofilm is a necessary constituent of periodontal illness and epigastric illness with *H. pylori* [15]. On the community level, the MDR become more numerous and have the capability to develop biofilm when foreign material is absent. Moreover, it has been noticed that community-associated MDR has the capability to infect healthy individuals if the immunocompromised individuals are not available. Immunity genes of the host develop specific polymorphisms that facilitate colonization of selected bacteria. In the case of the *Staphylococcus aureus* in nasal carriage, human genes have even been classified as the dominant decision [16].

The article "Multidrug-Resistant Bacteria: Their Mechanism of Action and Prophylaxis" was published in 2022. Journal: Biomed Res Int.

### 3.1. MRSA

The most common example of MDR bacteria is MRSA (methicillin-resistant *S. aureus*), i.e., transmitted efficiently from strict hospital-acquired infection to community-associated spread. However, the epidemiology of such CA-MRSA (community-associated methicillin-resistant *S. aureus*) has already been extensively evaluated [17, 18]. Numerous nonlactam antibiotics were found to be effective against such CA-MRSA strains. In the USA, a novel strain of CA-MRSA was discovered, i.e., known as the CA-MRSA-USA300 strain, that successfully substituted the previous USA400 CA-MRSA strain in the early 2000s [17]. It has been observed that this USA300 strain is distinguished by the existence of staphylococcal cassette chromosome mec (SCCmec) type IV along with the genes responsible for the secretion of Panton-Valentine leucocidin (PVL) toxins [19]. *P. aeruginosa* is well-known for causing nosocomial infections with symptoms such as pneumonia and bloodstream illness. Favorable environments for *P. aeruginosa* are moist places and can be found mostly in washing sinks, aerators, equipment like respiratory gear, and unhygienic solutions in the hospital environment [20]. Moreover, fewer patients have experienced the chronic biofilm-associated pseudomonal establishment along with cystic fibrosis (CF) [21]. Among such patients, repetitive applications of antibiotics lead to the origin of MDR bacterial strains. Community-associated infections with MDR strains of *P. aeruginosa* are found to be uncommon [22, 23]. In a group of 60 patients suffering from community-acquired bloodstream illness due to *P. aeruginosa*, 100% of isolates are meropenem susceptible, and 95% are susceptible to ceftazidime, tazobactam, and piperacillin [24].

### 3.2. Vancomycin-Resistant *Enterococci* (VRE)

One more antibiotic-resistant bacterial strain was developed in the late 1980s, i.e., VRE (vancomycin-resistant *Enterococci*), which is responsible for the major source of hospital-acquired infections in 1990. It has also become evident in the European study that such vancomycin-resistant *Enterococci* were isolated in the fecal material of healthy individuals [25]. Due to this variation between Europe and the USA, avoparcin is widely used. Avoparcin is a glycopeptide antibiotic, i.e., used to enhance the growth of animals as food additives. It has become evident that avoparcin was not permitted for use in the USA or Canada, but it was widely used in Europe until 1997 [26]. When the use of avoparcin was strictly prohibited in animal husbandry, the prevalence of vancomycin-resistant *Enterococci* was decreased in both animal samples and human volunteer samples [25, 26]. These examples show that there is a strong link between the use of antibiotics in food production and the rate of antimicrobial resistance in people.

The article "Multidrug-Resistant Bacteria: Their Mechanism of Action and Prophylaxis" was published in 2022. Journal: Biomed Res Int.

Afterwards, such VRE were collected from the wastewater from a semi-closed agri-food system [27]. However, VRE was found to be an unusual infectious agent among community-associated infections. Among the 289 individuals suffering from community-associated VRE, 85% of individuals undergo hospitalization, while 71% of individuals undergo antimicrobial contact within 3 months, respectively [28]. Moreover, conventional risk factors associated with antimicrobial exposure can be attained through serious infection, indwelling medical equipment, cancerous growth, and a weakened immune system [28, 29]. The increased prevalence of vancomycin-resistant *Enterococci* (VRE) in society is caused by either a constant influx of VRE into the food chain via shared community gut microbiome or increased antibiotic pressure. In terms of inducible resistance, the fitness costs of VRE for *Enterococci* were found to be almost nothing [30, 31].

It has been noticed that the majority of community-associated infections like UTI and bacteremia are mainly caused by members of the *Enterobacteriaceae*. Among the widespread ESBL groups (extended-spectrum beta-lactamases), 91% belong to the CTX-M group, while the rest are SHV (8%) and CMY-2 (1%). Among them, the majority of isolates (54%) belonged to the ST131 clonal group [32]. It has been observed that the community-onset infection by ESBL-producing *E. coli* is the most recurrent type, occurring mostly in Asia, the Middle East, South America, and a few regions of Europe. This infection, however, is less common in New Zealand, Northern Europe, and Australia. In such less frequently occurring areas, there is a particular risk factor associated with community-onset ESBL-producing *E. coli* infections. In a finding conducted in Australia and New Zealand, it was observed that individuals born in the Indian subcontinent or on a tour of India, China, Africa, or the Middle East were at high risk for community-onset third-generation cephalosporin-resistant *E. coli* infections [33].

Among Asian continents, an important issue is related to the dissemination of infection with *K. pneumoniae* strains. Such “hypermucoviscous” varieties have the tendency to develop community-onset pyogenic liver abscess along with metastatic illness and meningitis [34]. Such bacterial strains are mostly susceptible to a variety of antibiotics; community-onset ESBL-secreting strains are becoming more common [35]. Carbapenem is now the preferred drug recommended by physicians against the fatal infection of ESBL. Henceforth, the application of empiric carbapenem has improved remarkably to treat the widespread infection of such organisms within society.

The article "Multidrug-Resistant Bacteria: Their Mechanism of Action and Prophylaxis" was published in 2022. Journal: Biomed Res Int.

### 3.3. Carbapenem-Resistant *Acinetobacter baumannii* (CRAB)

*A. baumannii* is a Gram-negative bacillus that causes infections in hospitals and intensive care units [36]. Moreover, in Asia and Australia, the community associated with *A. baumannii* illness has been well-recognized [37]. In the majority of cases, such infections are coupled with pharyngeal carriage along with addiction to alcohol and smoking [37]. These infections are extremely lethal, accounting for approximately 56% of people suffering from bacteremia and/or pneumonia [37]. Certain natural resources like soil, fruits, and vegetables, along with animal and human skin and throat tissue, may serve as community reservoirs for *A. baumannii.* In addition to this, *A. baumannii* has also been isolated from human lice [38].

However, resistance to carbapenem may take place due to the accumulation of carbapenemases like IMP, associated oxacillinases (OXA), and carbapenemases [39]. The data of a study in Australia clearly reflects that out of 36 individuals suffering from community-onset bacteremic *A. pneumonia*, all were found vulnerable to carbapenems [40]. In another study in China, more troublesome results were obtained when out of 32 individuals suffering from community-acquired pneumonia caused by *A. baumannii*, and 3 and 6 isolates were nonsusceptible to meropenem and imipenem, respectively [41].

It has been noticed that *A. baumannii* having community-associated carbapenem-resistant infections is unusual and causes infection in natural habitats. It has become evident that carbapenem-resistant *Enterobacteriaceae* pose a serious threat to human health. From now on, immediate and timely action is required [1, 42]. In addition to it, carbapenem-resistant *E. coli* (CREC), i.e., an integral component of the CRE subset, was found to have a major epidemic in the USA [42, 43]. This CREC is not widespread in Asia, and such strains have been isolated from drinking water supplies in India and food-producing cattle in China [44].

But still, in such a populated country, people become afraid of the threat of CRE colonization [45, 46]. Moreover, much research data is available on carbapenemase-producing *E. coli* ST131 [47]. In India, research was conducted to compare the clinical isolates of ST131 with non-ST131. The findings of this study clearly showed that approximately 20% of clinical isolates tested positive for metallo-lactamases such as blaNDM-1, which was distributed evenly between ST131 and non-ST131 *E. coli* [48]. Moreover, it has been noticed that the distribution pattern of ESBL is found to be 10 years ahead of the carbapenemases. Henceforth, it is evident that community-associated carbapenem-resistant ST131 *E. coli* will pose a hazard in the near future.

The article "Multidrug-Resistant Bacteria: Their Mechanism of Action and Prophylaxis" was published in 2022. Journal: Biomed Res Int.

## 4. Antibiotic Resistance Mechanisms in Gram-Positive Bacteria

The major threat in the present scenario is an increase in MDR bacteria and the unavailability of novel antibiotics to kill them. Nowadays, the research is mainly focused on searching for novel methods to treat such MDR. In this direction, the major step has been laid down by the WHO by releasing a document containing the names of all deadly MDR which are resistant to all the available methods. Moreover, the WHO appeals to all nations to develop new novel drugs and other treatment methods to handle MDR successfully. In this document, certain Gram-positive bacteria like methicillin-resistant *Staphylococcus aureus*, drug-resistant *Streptococcus pneumonia*, vancomycin-resistant *Enterococcus faecium*, and many more are listed that pose a serious threat to societal health [1]. It has been noticed that such resistance develops in bacteria due to genetic mutations and/or acquired genomes [49] (Table 1).

It has been observed that a rise in the number of MDR is resulting in the nonavailability of any alternate to treat such strains, which henceforth is responsible for the high incidence of morbidity and mortality [50]. As discussed earlier, the WHO has drafted a list of such MDR and classifies them on the basis of severity of infection as medium, high, and critical antibiotic-resistant bacteria [51]. As per the WHO, there is an immediate requirement for some novel treatments against such MDR. Among such deadly pathogens, *β*-lactamase-resistant *Streptococcus pneumonia*, methicillin-resistant *Staphylococcus aureus* (MRSA), and vancomycin-resistant *Enterococcus faecium* (VRE) are major Gram-positive bacteria associated with multidrug resistance and posing a serious threat to society [1, 52]. There is some difference in the cell wall composition of Gram-positive and Gram-negative bacteria, as Gram-positive bacteria possess a thick layer of peptidoglycan over the cytoplasmic membrane that provides protection against adverse environmental conditions, and Gram-negative bacteria lack the LPS layer [53]. It is well-known that Gram-positive bacteria have mainly two basic morphologic forms, like cocci (e.g., *Staphylococcus*) and bacilli (e.g., *Bacillus*) [54]. Moreover, Gram-positive bacteria have teichoic acids, which are long anionic polymers, membrane proteins that make possible the incoming and outgoing of various molecules and capsular polysaccharides that are covalently linked to peptidoglycan [55]. There are two main mechanisms through which Gram-positive bacteria develop resistance to antibiotics. These are as follows:

- Secretion of *β*-lactamases, i.e., responsible for the enzymatic breakdown of antibiotics
- By reducing the affinity and susceptibility of their target site, e.g., PBP (penicillin-binding protein), through either attainment of exogenous DNA or through mutation among native PBP genes [56, 57]

Different antibiotics have diverse mechanisms of action. A few such examples are given below.

- Penicillin-binding proteins were targeted by *β*-lactams which bring about the end step of cell wall synthesis that ultimately cause cell death. *β*-lactamases are responsible for the deactivation of the antibiotic and hence develop resistance. The major source for the development of penicillin resistance takes place due to horizontal distribution of penicillinase plasmids through bacteriophages or through horizontal gene transfer which engage the genes for penicillin-binding proteins. In addition to this, methicillin resistance can develop from extra penicillin-binding proteins like PBP2/2a, i.e., obtained from foreign DNA elements [56–58]
- Vancomycin and teicoplanin are glycopeptides. These antibiotics also inhibit the end step of cell wall synthesis. Attainment of the van gene cluster (VanA, VanB, VanC, VanD, VanE, and VanG) is mainly responsible for the development of resistance that ultimately causes less binding affinity to glycoproteins [57–59]
- Other antibiotics like quinolones act on the DNA gyrase and topoisomerase IV enzymes and inhibit their function. This results in bacterial death. Resistance to quinolones develops due to the mutations occurring in the subunits of these two enzymes (grIA/grIB and gyrA/gyrB) [60, 61]
- Moreover, aminoglycosides have affinity for 30S ribosomal subunits that prevent the translocation process and hence produce nonfunctional proteins that upset the membrane structure and enhance aminoglycoside penetration. Resistance develops through the attainment of certain modifying enzymes like phophotransferases, nucleotidyltransferases, acetyltransferases, or through mutation and efflux mechanisms [62]
- On the other hand, macrolides have affinity for the 50S ribosome and prevent protein synthesis. Resistance developed as a result of various mechanisms such as mutations in the 23S rRNA and protein L4, methylation of the 23S rRNA, and efflux systems Mef (A) and Msr (A) [57, 63]
- Oxazolidinones, e.g., linezolid, have affinity for the 50S ribosome subunit and prevent protein synthesis. Resistance was achieved through mutations in 23S rRNA and G2576T in DNA [56, 64]

The article "Multidrug-Resistant Bacteria: Their Mechanism of Action and Prophylaxis" was published in 2022. Journal: Biomed Res Int.

### 4.1. Methicillin-Resistant *Staphylococcus aureus*

*Staphylococcus aureus* is Gram-positive cocci that belong to the *Staphylococcaceae* family. It is one of the major human pathogens responsible for fetal illness and increased mortality rates. It causes several deadly diseases, including infective endocarditis, skin, respiratory tract, and soft tissue infections, and infections of pleuro-pulmonary-related devices [65, 66]. It also has a high level of resistance to several antibiotics. Penicillin-resistant *S. aureus* secretes a plasmid-mediated penicillinase, which breaks the *β*-lactam ring of penicillin, which is required for its antimicrobial activity [67]. Celbenin, now known as methicillin, is a derivative of penicillin and was introduced to neutralize the bacterial resistance mechanism. Resistance develops as a result of the production of extra penicillin-binding proteins like PBP2a, which reduces the affinity for penicillin and *β*-lactam antibiotics [65, 68, 69].

### 4.2. Vancomycin Intermediate and Resistant *Staphylococcus aureus*

MRSA is a deadly pathogenic MDR, and it has been noticed that VISA and VRSA have originated from MRSA itself. Due to variation among the resistance mechanisms, VRSA does not develop into VISA. Vancomycin kills the bacterial cell by breaking the PPCB (pentapeptide cross bridge) bond between two NAM units (D-Ala-D-Ala residues) [70, 71]. It is well-known that the cell walls of Gram-positive bacteria are very thick. Henceforth, these D-Ala-D-Ala residues serve as decoy targets in the thickened cell wall and block vancomycin on the outer surface of the cell wall, causing misreading in identifying its true targets. Moreover, VRSA attained this genetic resistance from vancomycin-resistant *Enterococci* (VRE). Until now, six VRSA strains have been isolated and characterized in the USA, and each one has attained the vanA genes, i.e., the genes responsible for providing a high degree of resistance to teicoplanin, glycopeptides, and vancomycin. It has been noticed that VanA genes are responsible for the manufacturing of modified peptidoglycan precursors having a terminal D-Ala-D-Lac, where vancomycin reflects much less affinity in comparison to the terminal wild-type D-Ala-D-Ala [69] (Figure 1).

The article "Multidrug-Resistant Bacteria: Their Mechanism of Action and Prophylaxis" was published in 2022. Journal: Biomed Res Int.

### 4.3. Ampicillin/Penicillin and Cephalosporin Resistance *Enterococcus faecium: faecium*

*E. faecium* is Gram-positive cocci from the *Enterococaceae* family*. E. faecium* develops resistance against *β*-lactams, e.g. penicillin, as it is linked with the pbp5 chromosomal gene, i.e., responsible for the secretion of a low binding affinity class B PBP for ampicillin/penicillin and the cephalosporins. In addition, mutations in penicillin-binding proteins and hypersecretion of *β*-lactamase enzymes lead to the development of resistance to *β*-lactam antibiotics. Furthermore, other mechanisms are found to be associated with the resistance to cephalosporins as they undergo similar types of response regulator, CroR, serine/threonine kinase designated IreK, and phosphatase IreP [72, 73].

### 4.4. *E. faecium* (Vancomycin-Resistant)

*E. faecium* is a Gram-positive bacterium that attained special genes that are present in the plasmid (extra chromosomal DNA), which were classified into 6 of the 19 families and transposons like Tn1547 that provide resistance to vancomycin [74]. Vancomycin, like penicillin, binds to the D-alanyl-D-alanine (D-Ala-D-Ala) terminus and inhibits cell wall synthesis. It has been observed that gene clusters responsible for vancomycin resistance like van A, B, D, and M carry out the substitution of D-Ala-D-Ala by D-alanyl-D-lactate termini which, i.e., are accountable for the low binding affinity of vancomycin. Among them, the Van A gene cluster was discovered to be the most effective and to be present on a transposon, i.e., linked to Tn1546 [75].

#### 4.4.1. Other Mechanisms of Resistance

As already discussed, fecal resistance to vancomycin is widespread. Moreover, this bacterium also has resistance to aminoglycosides such as gentamicin, tobramycin, and kanamycin because it poses aminoglycoside-modifying enzymes (AMEs) containing aminoglycoside nucleotidyltransferases (ANTs), aminoglycoside acetyltransferases (AACs), and aminoglycoside phosphotransferases (APHs). In addition to that, attainment of genes responsible for encoding ANT(3”)-Ia or ANT(6)-Ia enzymes along with mutation in S12 ribosomal protein develops a high degree of resistance against streptomycin. Besides it, *E. faecium* also reflects strong resistance to fluoroquinolones through making point mutations in gyrA and parC genes, i.e., those responsible for the encoding subunits A of and topoisomerase IV or DNA gyrase or NorA-like efflux pump. Additionally, *E. faecium* also reflects resistance to quinupristin–dalfopristin (a streptogramin drug) that inhibits bacterial protein synthesis through binding to 23-S rRNA of the 50S ribosomal subunit and stops its function [76].

The article "Multidrug-Resistant Bacteria: Their Mechanism of Action and Prophylaxis" was published in 2022. Journal: Biomed Res Int.

### 4.5. *Streptococcus pneumoniae* (Penicillin-Nonsusceptible)

Among Gram-positive bacteria, the most common pathogenic bacteria is *S. pneumonia*, which adheres to the upper respiratory tract and is capable of causing infections such as pneumonia, meningitis, bronchitis, and sinusitis. It reflects penicillin resistance by causing changes in one or more of the six penicillin-binding proteins found in its cell membrane. This occurs because of chromosomal mutations or may be attributed to the usual transformation process in which the DNA is taken up from other bacteria and is inserted inside the *Pneumococci* (host) DNA. This *Pneumococci* is capable of causing infection in older people. Children and daycare workers are more prone to this resistant *Pneumococci* infection [77, 78]. Moreover, *Pneumococci* not only undergo resistance to penicillin but also to erythromycin and trimethoprim-sulfamethoxazole (TMP-SMX). Furthermore, the erm(B) gene, which is responsible for methylase secretion, is responsible for resistance to macrolide-lincosamide-streptogramin B. Similarly, the mef(A) gene also undergoes similar resistance through an antibiotic efflux pump. Some other mechanisms for resistance have also been noticed, which include mutations in ribosomal proteins L4 and L22 leading to the dysfunction of ribosomal RNA (23S rRNA). Antibiotic resistance was also discovered against fluoroquinolones, tetracyclines, and chloramphenicol [79, 80].

### 4.6. Other Resistant Gram-Positive Bacteria and their Resistant Mechanisms

The tendency to develop biofilms and the presence of exopolysaccharide matrix are a few mechanisms that develop resistance in *Staphylococcus epidermidis* through decreasing penetration and diffusion of antibiotics. *S. epidermidis* is primarily responsible for hospital-acquired infections due to the transport of resistant mecA genes that encode PBP2a. Moreover, they also show resistance to vancomycin and quinolones [81]. The major cause of uncomplicated UTIs (urinary tract infections) is caused by *Staphylococcus saprophyticus.* This bacterium undergoes resistance against several antibiotics like ciprofloxacin, ampicillin, cephalexin, and ceftriaxone [82].

The most common commensal bacterium, *Streptococcus viridians*, which lives in the human upper respiratory tract, develops resistance to antibiotics such as penicillin and other *β*-lactam drugs by modifying the penicillin-binding protein. In a few studies, it has been mentioned that *S. viridans* act as reservoirs for resistance genes like mef (E) and mel genes that show resistance to macrolide-lincosamide-streptogramin B (MLS (B)) antibiotics [83, 84]. Another bacterial pathogen that is established in the upper respiratory tract and skin is *Streptococcus pyogenes* that shows resistance against streptogramins, macrolides, and lincosamides. Moreover, it also reflects resistance to aminoglycosides, fluoroquinolones, and tetracyclines [85]. It has been noticed that most neonatal infections in humans are caused by *Streptococcus agalactiae* or group B *Streptococcus* (GBS), i.e., Gram-positive cocci. During delivery, this pathogen might be transformed from mother to baby. Resistance to erythromycin and other macrolides occurs in *S. agalactiae* via changes in ribosomal function, mediated by erm genes, or via efflux pumps encoded by mefA genes. Apart from this, linB genes are responsible for inhibiting the ribosomal translocation that develops clindamycin resistance in GBS [86].

The article "Multidrug-Resistant Bacteria: Their Mechanism of Action and Prophylaxis" was published in 2022. Journal: Biomed Res Int.

## 5. Gram-Negative Bacterial Resistance to Antibacterial Agents and Methods to Overcome It

Natural products have been used to cure many ailments since ancient times. For example, the cinchona tree contains quinine, which is used to treat malaria. Since Fleming discovered penicillin in 1929, a plethora of antibacterial medicines have been developed, all of which have had a significant influence on human health and death rates across the world [87]. Antibiotics have been overused and misused, resulting in the emergence of new resistant forms. People in impoverished nations can readily obtain antibiotics without a prescription, so public awareness of the issue is critical [88]. Bacteria can evade antibiotics by a variety of processes, including neutralizing antibiotics, pumping them outside the cell, or altering their outer structure, resulting in drug inhibition. All of these strategies lead to the evolution of antibiotic resistance in bacteria. There are four types of antibiotic resistance mechanisms in bacteria: intrinsic resistance, where bacteria modify their structure and components, and acquired resistance, when bacteria acquire new resistant genes or DNA from other bacteria. Additionally, certain genetic alterations in the gene can result in protein modifications, resulting in new components and receptors for antibiotics to identify, and lastly, DNA is transmitted across bacteria by combination, transduction, or transformation [53].

We employ the complex formed by the addition of crystal violet-iodine followed by safranin as a counter stain to discriminate between Gram-positive and Gram-negative bacteria, as developed by Christian Gram. Gram-positive bacteria keep their complex stain and look purple, but Gram-negative bacteria lose their complex stain and appear pink owing to counter stain. The change in cell wall composition between two species of bacteria is the cause of this discrepancy [87, 88]. Three layers make up the envelope carried by Gram-negative bacteria. The outer membrane, which serves as a protective barrier, has a unique characteristic that distinguishes Gram-positive bacteria from Gram-negative bacteria. Lipo-polysaccharides are bound in the inner leaflets of the outer membrane, whereas phospholipids are bound in the outer leaflets. Furthermore, the outer membrane contains proteins such as porins and others that enable diverse molecules to flow through it (Figure 1). The bacterial cell wall, i.e., composed of peptidoglycan, is made up of repeating units of NAM and NAG, which help in regulating the cell shape [53]. The second layer, discovered in the subsequent layer, the inner membrane, is composed of phospholipids that serve various roles, including structure, biosynthesis, and transport. It also serves as a location for DNA anchoring and aids in the separation of sister chromosomes [89].

The article "Multidrug-Resistant Bacteria: Their Mechanism of Action and Prophylaxis" was published in 2022. Journal: Biomed Res Int.

Antibiotic resistance has been linked to the outer membrane of bacteria, which includes *β*-lactase, quinilons, colistins, and other antibiotics. Antibiotics must be able to pass through the cell wall to reach the target, much as hydrophilic medications can pass via porins and hydrophobic drugs may pass through diffusion. Any change or mutation in the outer membrane can lead to the development of resistance. Gram-negative bacteria become more antibiotic resistant than Gram-positive bacteria because Gram-positive bacteria lack this layer [90, 91]. Gram-negative bacteria are frequently observed causing illness in humans, particularly in immunocompromised people. Due to resistance, Gram-negative bacteria produce the most difficult nosocomial infections [92]. Antibiotic inactivating enzymes are the main cause of antibiotic resistance in Gram-negative bacteria, which can be acquired by plasmids, aminoglycoside-modifying enzymes, or other mobile genetic elements carrying resistance genes or as a result of increasing intrinsic resistance due to mutations in chromosomal genes. A nonenzymatic pathway for fluoroquinolone resistance among *Enterobacteriaceae* was also observed, such as a plasmid-borne quinolone resistance gene [93].

### 5.1. Cephalosporin of the Third Generation for *Enterobacteriaceae*

The synthesis of beta-lactamses by resistant *Enterobacteriaceae* causes resistance to third-generation cephalosporins. ESBLs, for example, can hydrolyze broad-spectrum cephalosporin monobactams and penicillins. Resistance to early generation cephalosporins, ampicillin, and amoxicillin is caused by class A beta-lactamase such as SHV-1, TEM-1, and TEM-2. Resistance to third-generation cephalosporins develops when mutations in genes encoding TEM-2, TEM-1, or SHV-1 produce novel beta-lactams capable of hydrolyzing them. Carbapenem-resistant bacteria CRE is an *Enterobacteriaceae* isolate that is resistant to all carbapenem antimicrobials, including ertapenem, imipenem, and meropenem. Due to the synthesis of AmpC beta-lactamases and the loss of outer membrane protein, the initial isolates developed resistance. Carbapenem-producing CRE (CP-CRE), whose genes are found on mobile genetic elements, and noncarbapenem-producing CRE (non-CP-CRE) are the two forms of CRE that are generally recognized [12]. The following are the five main carbapenemases:

- OXA-48, a carbapenemase-like class D OXA
- Pneumocystis pneumonia
- New Delhi metallo-lactamases, class B (NDM)
- Metallo-lactamases encoded by Verona integrin (VIM)
- On imipenem, IMP is active. *Morganella morganii*, *Proteus* spp., and *Providencia* spp. are among the *Enterobacteriaceae species* with inherent imipenem resistance [94]

The article "Multidrug-Resistant Bacteria: Their Mechanism of Action and Prophylaxis" was published in 2022. Journal: Biomed Res Int.

### 5.2. *Acinetobacter baumannii*

*A. baumannii* is a Gram-negative bacterium that is aerobic in nature and is one of the most dangerous species among *Enterococcus faecium*, *Staphylococcus aureus*, *Klebsiella pneumoniae*, *Pseudomonas aeruginosa*, and *Enterobacter species* (*ESKAPE*) declared by the WHO to be capable of neutralizing antibiotic effects [95]. *A. baumannii* has also been linked to nosocomial infections all over the world.

Mechanisms via which it can acquire antibiotic resistance quickly:

- The inactivation of beta-lactams by beta-lactamases is a common MDR mechanism. *A. baumannii* has demonstrated that all four *β*-lactam classes, A, B, C, and D, can integrate foreign DNA into their genomes and can quickly recognize a large number of *β*-lactams. Some of these enzymes are narrow-spectrum beta-lactamases, whereas others are involved in ESBL hydrolysis, which can reduce carbapenem sensitivity
- Multidrug efflux pumps, which are resistant to a variety of antibiotics, including imipenem, are another source of resistance in *A. baumannii*. The four recognized types of efflux pumps are multidrug and toxic compound extrusion (MATE), resistance nodulation division (RND) superfamily, major facilitator superfamily (MFS), and small multidrug resistance (SMR) family transporters [95]
- The three types of enzymes present, acetyltransferases, adenyltransferases, and phosphotransferases, are important in mediating *A*. *baumannii's* resistance to aminoglycosides. These enzymes change the chemical structure of aminoglycosides. Coding genes can be transferred by transposons, integrons, and plasmids
- Changes in the envelope's permeability have an impact. Porins, which are proteins, are found in the outer membrane and form channels that allow molecules to pass through. This is a crucial part of the resistance process. Some porins, such as Caro and Omp22-33, have been linked to carbapenem resistance in *A*. *baumannii*

The article "Multidrug-Resistant Bacteria: Their Mechanism of Action and Prophylaxis" was published in 2022. Journal: Biomed Res Int.

### 5.3. *Pseudomonas aeruginosa*

*Pseudomonas aeruginosa* is one of the most dangerous pathogens in the ESKAPE group. It is a Gram-negative bacterium that is present in the typical flora of the intestine. In critically unwell patients, it is also responsible for ICU-acquired infections. Innate resistance mechanisms, such as overexpression of the efflux pump and decreased permeability of the outer membrane, as well as acquired resistance mechanisms, such as the acquisition of resistance genes and mutations in genes that encode for proteins called porins and other proteins, can make this bacterium difficult to treat. Antibiotics like penicillin, carbapenem, and cephalosporin disrupt the bacterial peptidoglycan cell wall production. Ceftazidime and cefepime, which belong to the third and fourth generations of cephalosporins, are two of the most effective *β*-lactams for treating *Pseudomonas aeruginosa* [96].

*β*-lactamases break the amide link in the beta-lactam ring, rendering medicines ineffective. A, B, C, and D are the four primary classes of *β*-lactamases discovered in *Pseudomonas aeruginosa*. The enzymatic activity of serine residues suppresses *β*-lactams in classes A, C, and D, whereas zinc cation is required for class B's effect. *Pseudomonas aeruginosa* can also gain resistance by gene mutation, which can result in AmpC *β*-lactamase overexpression. Amp G encodes for a transmembrane protein that works as an A permease for 1,6-anhydromurapeptides that induce ampC, while amp D eventually encodes for a cytosolic N-acetyl-anhydromuramyl-L-alanine amidase that acts as an abridge for Amp C production.

*Pseudomonas* resistance to aminoglycosides is caused by transferable aminoglycoside-modifying enzymes. These enzymes are divided into three groups: aminoglycoside acetyltransferases (AAC), aminoglycoside phosphoryl transferases (APHs), and aminoglycoside adenylyl transferases (AADs). They are able to inactivate aminoglycosides by joining a phosphate, adenyl, or acetyl radical to the present antibiotic molecule, reducing their ability to bind with their target in the bacterial cell. Besides beta-lactams, colistine has been reported to be more effective against MDR *Pseudomonas* when combined with an anti-*Pseudomonas* medication such as ceftazidime, ciprofloxacin, or imipenem. Fosfomycin therapy in combination with aminoglycosides, cephalosporins, and penicillins has also been shown to be effective in the treatment of MDR *Pseudomonas aeruginosa* [96].

The article "Multidrug-Resistant Bacteria: Their Mechanism of Action and Prophylaxis" was published in 2022. Journal: Biomed Res Int.

### 5.4. *Helicobacter pylori*-Clavithromycin-Resistant

*Helicobacter pylorus* is a Gram-negative bacterium that has been identified as one of the most significant pathogens in humans, causing gastritis, peptic ulcers, and stomach cancer. It has been stated that the efficacy of *Helicobacter pylori* is increased as a result of the rapid development of resistance to antibiotic therapy, and therefore, the treatment efficiency is reduced [97, 98]. Overexpression of efflux and the translation initiation factor IF-2 with ribosomal protein L22 have also been linked to the development of resistance.

### 5.5. Fluoroquinolone Resistance in *Salmonella* spp.

Bacteria that are Gram-negative Salmonellae are split into two types: typhoidal *Salmonella* and nontyphoidal *Salmonella*, both of which are pathogenic to humans. MDR in *Salmonella* has been documented against ampicillin, chloramphenicol, and sulfamethoxazole, prompting the use of FQ-ciprofloxacin and ceftriaxone, the third generation of cephalosporins, which has resulted in the fast development of resistance to these medications. This has been cited as one of the main reasons for the World Health Organization's designation of FQ-resistant *Salmonella* as an important pathogen for research and development of novel antibiotics in 2017. Mutations in the quinolone resistance determining areas of the chromosomal gyr and par genes have been shown to cause quinolone resistance. As a result of this, quinolone has poor binding affinity for topoisomerase enzymes. Another method worth mentioning is plasmid-mediated quinolone resistance (PMQR), where physical protection is supplied by genes like Qnr, the Aac-60-lbcr gene reduces FQ action, and quinolone efflux pumps are encoded by oqxAB and qepA [99].

## 6. Alternative Techniques for Controlling MDR Infections

### 6.1. Use of Nanotechnology to Create anti-MDR-Resistant Nanobacterial Agents

According to one study, nanoparticles can be used to replace antibiotics and certain disinfectants. Liposome nanoparticles made of both inorganic and organic materials, such as silver, zinc, gold, and copper, can be used as antibiotics and disinfectants. The majority of examples of nanoparticles being used as antibiotics include preventing catheter-associated urinary tract infection (CAUTI) and biofilm development. Nanoparticles have also been used in antibacterial wound dressings and coatings [100–106]. Antimicrobial resistance to a therapeutic treatment in bacterial pathogens is not difficult to develop, as resistance can be generated even through basic genetic changes and modifications [107]. The antibiotic combinatorial method is thus one of the most promising strategies for limiting antimicrobial resistance [108].

The article "Multidrug-Resistant Bacteria: Their Mechanism of Action and Prophylaxis" was published in 2022. Journal: Biomed Res Int.

Nanodelivery systems increase the vulnerability of MDR bacterial strains to specific antibiotics by protecting them from bacterial hydrolytic enzymes and suppressing resistance mechanisms such as changes in outer membrane porin proteins that result in antibiotic impermeability [109]. Individual nanoantibiotic complexes have different working procedures and configurations than individual antibiotics. When nanoparticles are conjugated to therapeutic drugs like antibiotics, a synergistic antibacterial effect may be obtained; they can also create nanocarrier antimicrobial complexes with bactericide properties [110]. Antimicrobial agents that are unstable, such as bacteriophages, phytochemicals, peptides, and antibiotics, can be delivered by utilizing both organic and inorganic materials, such as chitosan and gold nanocarrier systems and drug nanovectors [111]. In an experiment [112], pomegranate ring extract (PGRE) has also been shown to inhibit the release of bacterial flagellins.

The restoration of the chemicals inside the nanohybrid has been documented in both experiments. The polyelectrolyte (PAH) surface-modified gold nanoparticles and silver nanoparticles had a symbiotic repressive effect of about 100% on Bacillus Calmette-Guerin and *E. coli* [113], while the silver nanoparticles conjugated with curcumin had a combined antimicrobial effect on *Pseudomonas aeruginosa* and *E. coli* [114]. In rat models, monotype chemoattractant protein-1 (MCP-1) nanocoated on orthopedic implants with interleukin-12 p70 (IL-12p70) and multilayer polypeptide nanoscale coatings with IL-12 [115] powerfully arouse the body's innate defense against open fracture [116]. In another investigation, a ceragenin-coated iron oxide magnetic nanoparticles (MNP CSA-13) hybrid was created. Despite its significant antibacterial action, ceragenin (CSA-13), a synthetic peptide, has been restricted in usage because of its nonselective toxicity.

At extremely high concentrations of around 100 micrograms/ml, the MNP-CSA-13 nanocomposite produced by conjugating iron oxide magnetic nanoparticles (MNP) with CSA-13 apparently targets primarily *P. aeruginosa* biofilms and free live cells. The absence of erythrocyte hemolysis indicates that conjugating synthetic peptides with nanocarriers reduces host cytotoxicity [117]. Glutaraldehyde [118] was used to establish a relationship between MNPs and CSA-13. The functional amino terminal silica on MNPs' surface was created by reacting glutaraldehyde with 3-aminopropyl trimethoxy silane (APTMS). CSA-13 binds to the MNP surface's terminal aldehyde groups, which react with CSA-13's main amine groups. MNP-CSA-13 may become dissociated at low pH due to inflammation and infection. Due to the hydrolysis of the imine link at low pH, the MNP-CSA-13 nanocomplex dissociates, and the CSA-13 antimicrobial peptide is liberated. As a result, the MNP-CSA-13 nanocomplex offers a promising nanodrug vector for pH-dependent standard antimicrobial administration to kill bacteria at infection sites where the pH is less than six [119].

The article "Multidrug-Resistant Bacteria: Their Mechanism of Action and Prophylaxis" was published in 2022. Journal: Biomed Res Int.

#### 6.1.1. Nanoparticles' Efficacy against Bacterial Biofilms and Spores

Because bacterial biofilms enable the conjugation of plasmids containing antibiotic genes and the biofilm matrix protects bacterial cells in lower films from antibiotics, assertions that bacterial biofilms are extremely tolerant and resistant to antibiotics [120] have been made. Organic and inorganic nano-ordered surfaces and coatings are now the most popular alternatives for preventing biofilm growth on medical devices [121]. The experiments of [122, 123] show that zeolitic imidazolate framework (ZIF), nanodragger arrays, and nanostructured polyurethane can prevent the formation of *Staphylococcus epidermis*, *S. aureus*, *E. coli*, and *P. mirabilis* biofilms by allowing bacterial cells to adhere to the topography of the nanolayered surface.

### 6.2. Essential Oils and Mono-/Bi-/Tri-Metallic Nanocomposites as Alternate Sources of Antibacterial Agents in the Fight against Multidrug-Resistant Pathogenic Microorganisms

Plants' active phytochemicals, bioactive substances, secondary metabolites, and essential oils are thought to be important in combating antibiotic resistance in pathogenic bacteria. Some alternative antimicrobial medicines can help to slow the spread and development of resistance to certain diseases. Essential oils are natural substances made up of volatile secondary metabolites extracted from various parts of plants, including flowers, seeds, buds, twigs, leaves, barks, herbs, roots, and fruits [124, 125]. Some of the most common chemical constituents of essential oils are flavonols, flavonoids, phenols, terpenoids, polyphenols, tannins, quinones, flavons, coumarins, alkaloids, lectins, and polypeptides, which have potential biological activities such as antioxidants, insecticidal, antiseptic, antiallergic, anti-inflammatory, antiviral, or antimicrobial properties. Many plants' essential oils are utilized in aromatherapy, food flavoring and additives, cosmetics, polymers and resins, and perfumes [126]. Many essential oil components have antibacterial characteristics, with terpenes including carvacrol, geraniol, menthol, and thymol having the strongest antimicrobial qualities.

The article "Multidrug-Resistant Bacteria: Their Mechanism of Action and Prophylaxis" was published in 2022. Journal: Biomed Res Int.

Essential oils have a wide spectrum of inhibitory actions against many bacterial pathogens [127], since they may readily enter the lipid component of the bacterial cell membrane and break the cell wall structure [128]. The loss of integrity and cellular content caused by the combination of essential oils and lipids leads to cell death [129]. Few essential oil components, such as terpene-4-ol terpenol isomers, inhibit cellular respiration and render the cell membrane ineffective as a permeable barrier [130, 131]. The amount of bioactive components found in various essential oils, for example, has a significant and unique function; essential oils isolated from cinnamon and black pepper, for example, damage cell membranes and inhibit *E. coli* and *S. aureus* metabolic activity [132, 133]. Another example is *Dipterocarpus gracious* essential oil, which inhibits the development of *P. mirabilis* and *B. cereus* by infecting their cytoplasm membrane. Essential oils acquired from *Lawsonia inermis*, *Zanthophylum alatum*, *Ammodaucus leucotrichus*, *Marrubium globosum*, *Citrus sinensis*, and *Zanthophylum alatum* have shown significant antioxidant activity along with *Menta spicata* L. and *Eremanthus erythropappus* M [134–139].

#### 6.2.1. Metallic Nanoparticles with Antimicrobial Properties

Aluminum oxide, iron oxide, titanium dioxide, copper oxide, zinc oxide, nickel oxide, zirconium dioxide, and chromium oxide nanoparticles have all been shown to have antibacterial properties. Metal and metal oxide base nanoparticles bind to the cell membrane, releasing metallic ions into the bacterial cell wall's proteins and enzymes. In addition, nanoparticles can harm the bacterial cell wall in a variety of ways, including electrostatic attraction, Van der Waals forces, and hydrophobic interactions [140–142].

#### 6.2.2. Essential Oil Nanoencapsulation Efficiency

Capturing essential oils in innovative nano-based delivery systems such as nanoemulsions, microemulsions, solid lipid nanoparticles, and liposomes are examples of how natural bioactive substances may be encapsulated to boost antibacterial activity. As nanoemulsions, lime essential oils encapsulated with chitosan showed enhanced antibacterial activity against *S. aureus*, *L. monocytogenes*, *Shigilla dysenterias*, and *E. coli* [143, 144]. *Aspergillus parasiticus* and *Schinus Moller* use chitosan [145, 146], lipid phase, and orecirol as solid lipid nanoparticles against *Aspergillus flavus*, *Aspergillus niger*, *Aspergillus ochraceus*, *Alternaria solani*, *Rhizopus stolonifer*, and *Rhizoctonia solani* [147]. Furthermore, chitosan with cardamom essential oil as nanoencapsulation against *S. aureus* and *E. coli* [148], chitosan with cardamom essential oil as nanocomposites against *S. aureus* and *E. coli* [149], and *Siparuna guianensis* with chitosan as nanoencapsulation against *Aedes aegypti* as nanoencapsulation [150].

The article "Multidrug-Resistant Bacteria: Their Mechanism of Action and Prophylaxis" was published in 2022. Journal: Biomed Res Int.

### 6.3. Nonribosomal Antibacterial Peptides (NRAPs) That Target Multidrug-Resistant Bacteria

NRAPs are a subclass of nonribosomal peptides that are produced by gigantic nonribosomal peptide synthetases (NRPSs) [151]. The NRPSs are made up of several modular sections, each of which is in charge of fusing amino acids into peptide-like products [152, 153]. The variable biosynthetic pathway of NRAPs results in the formation of molecules with structural diversity.

The rapid advancement of DNA sequencing technology has aided genomic data availability. Bioinformatics tools like NRPS Predictor 2, 122, Minowal 123, and PRISM 121 [154] may be used to identify and study possible BGCs from stored genomic sequences. These are frequently used, publicly accessible algorithms for predicting genetically encoded NRPs, such as PRISM, which predicted a cyclic telomycin derived from *Streptomyces canus* by mining biosynthetic scaffolds and characterized it with a novel antibacterial action by targeting cardiolipin [155]. Humimycin was also created via solid phase peptide synthesis, which is based on the investigation of the human microbiome using bioinformatics techniques and has a novel antibacterial action that targets lipid II lipase in MRSA and other bacteria [156].

The NRAP of baecaucein without lipid modification has demonstrated specific antibacterial action against MRSA in both *in vivo* and *in vitro* settings. Baecaucein-1 has all L-type amino acids, and the cationic guanodino group plays a major role in its action under physiological conditions, suggesting that the design of a linear peptide can be utilized as a basis for next-generation antibiotics [157]. The shortest known natural tripeptide with antibacterial action has been discovered [158], and the NRAP makes them more accessible.

## Figures and Tables

**Figure 1:** Resistance mechanisms found in Gram-positive and Gram-negative bacteria.

**Table 1:** Mechanism of antibiotic resistance.

S. No.	Kind of antibiotic resistance	Mechanism involved in resistance
1	*Restricting entry of antibiotics*	Antibiotics spread out in the cell through the occurrence of mutations in the gene which specifically encodes the outer membrane porin protein, and this results in the change in OMPK36 variant porin which shows less permeability for the antibiotics in *Klebsiella pneumonia* [159]. Because of the downregulation of the main porin protein or refilling the cell membrane with some another selected protein channel, the permeability of membrane for antibiotics in some bacteria such as *E. coli* and *Acinetobacter* is decreased [160].
2	*Accession of various efflux pump genes related to chromosomal and plasmid*	Through strong efflux pumping, the numbers of antimicrobials are launched out of the cell. Their overexpression allows resistance to formerly effective antibiotics example—MDR efflux pump in *Pseudomonas aeruginosa* and *E. coli* [161].
3	*Moderation and defense of antibiotic target*	By changing the arrangement of the targets, the binding affinity of antibiotics can be reduced. *Klebsiella pneumonia* and *Staphylococcus aureus* are found to be resistant to linezolid, and this is achieved by the mutation in allele which encodes the 23 s rRNA ribosomal subunit [162]. Development of resistance to the certain drugs such as macrolids, lincosamines, and streptograminscan be attained by doing methylation of their binding site and the 16 s rRNA by the action of enzyme called erythromycin ribosomal methylase and family. Resistance to the several other group of drugs such as penicillin, pleuromutilins, lincosamides, and oxazolidons can be achieved with the help of enzyme chloramphenicol florfenicol resistance methyltransferase through the incorporation of CH_3_ to A2503 in the 23 s rRNA [163]. Resistance to methicillin in *S. aureus* is because of the genetic discovery of chromosomal mec A which records a single binding protein for extra penicillin, PBP2a, with a less affinity for all *β*-lactam [164].
4	*Antibiotic opposition via hydrolytic enzymes*	The resistance is achieved by chromosomal detection, and plasmid-mediated encoding genetic enzyme degrades with antibiotics, for example, *β*-lactamase which includes penicillinase only degrading penicillin, cephalosporinases deactivate cephalosporins and aminopenicillins, and expanded beta-lactamases, which play an important role in digesting all *β*-lactam, but carbapenemase and carbapenem disabled the whole *β*-lactamase [165].
5	*Moderation of antibiotic resistance*	Detection of gene enzymes is deactivated by antibiotics with the addition of an active functional group. For instance, resistance to aminoglycolides in *Campylobacter coli* (*C. coli*) that is microaerophilic Gram-negative bacteria is caused by nucleotidylation, acetylation, and phosphorylation of its -OH and CO-NH groups by acetyl transferases, phosphotransferases, and nucleotidyltransferases [166].
